RETRACTED

# Clinical Study of Virtual Reality Augmented Technology Combined with Contrast-Enhanced Ultrasound in the Assessment of Thyroid Cancer

**DOI:** 10.1155/2021/8042755

**Published:** 2021-08-06

**Authors:** Qinghua Liu, Jian Cheng, Jingjing Li, Lei Liu, Hongbo Li

**Affiliations:** ^1^Ultrasonography Department, Rizhao People's Hospital, Rizhao 276826, Shandong, China; ^2^General Surgery, Rizhao People's Hospital, Rizhao 276826, Shandong, China

## Abstract

Thyroid cancer has become the most common malignant tumor in the endocrine system, and its global incidence has been showing an upward trend. The diagnosis methods of thyroid cancer include ultrasound, fine-needle aspiration cytology, and neck CT, but the single ultrasound feature cannot simultaneously take into account the sensitivity and specificity of more than 85% when diagnosing thyroid cancer. The development of virtual technology can significantly improve the diagnosis of the thyroid gland. Based on this, this article proposes a clinical study of virtual reality technology combined with contrast-enhanced ultrasound in the assessment of thyroid cancer. This article uses a variety of methods, such as literature method, mathematical statistics, and experimental research, in-depth study of the theoretical cornerstones of virtual reality augmented technology, the application status of ultrasound contrast technology, and so on. And a fuzzy mean clustering algorithm was proposed to identify ultrasound images. Then, a clinical experiment of virtual reality augmented technology combined with contrast-enhanced ultrasound was designed to evaluate thyroid cancer, which included comparison of contrast-enhanced ultrasound signs, analysis of enhancement results, multifactor logistic analysis, and diagnostic efficacy analysis of ultrasound signs. The combined application of virtual reality augmented technology and contrast-enhanced ultrasound in the study of thyroid cancer has a sensitivity and specificity exceeding 85% as the diagnosis boundary changes, and the accuracy of the combined diagnosis is relatively high.

## 1. Introduction

Thyroid cancer (TC) is a common endocrine malignant tumor. As we all know, the incidence of TC has been increasing significantly in recent years. Since almost all TCs require surgical treatment, the proportion of thyroid surgery is also on the rise. At the same time, a number of TC management guidelines at home and abroad have been revised several times, and their treatment methods have gradually become conservative. Since then, many scholars have summarized and evaluated the changing trends of TC's incidence, clinicopathological characteristics, treatment methods, and prognostic outcomes. In my country, the diversification of TC surgical methods, due to the irregular scope of surgery in the early years, has gradually become standardized and unified since the release of China's differentiated thyroid cancer (DTC) management guidelines in 2012. At present, the guidelines and the 2015 American Thyroid Association (ATA) guidelines have become an important evidence-based medicine basis for the diagnosis and treatment of TC in my country. This shows that the surgical methods of TC have changed, but there is no systematic report on the surgical changes of TC and related influencing factors in China.

RETRACTED

Contrast-enhanced ultrasound harmonic imaging technology significantly improves the contrast between the contrasted area and adjacent tissues [1] and is also called noninvasive microcirculation angiography [2]. This technology can provide early detection of tumor microcirculation perfusion characteristics to identify benign and malignant and small tumors or evaluate the tumor residue after interventional treatment, locate vascular stenosis, occlusion, deformity, and traumatic bleeding caused by trauma, and understand the degree of bleeding for further treatment [3, 4]. Contrast-enhanced ultrasound has been widely used in the differentiation of benign and malignant tumors, such as the liver, kidney, pancreas, spleen, and prostate.

Thyroid cancer is the most common endocrine malignancy. There are two subtypes of thyroid cancer (DTC), papillary thyroid cancer (PTC) and follicular thyroid cancer (FTC), which are the most common subtypes of thyroid cancer. Medullary thyroid cancer (MTC) and anaplastic thyroid cancer (ATC) are even rarer. In recent years, the incidence of DTC has increased rapidly due to the more frequent use of imaging methods such as neck ultrasound and fine-needle aspiration (FNA) of thyroid nodules. After total thyroidectomy and radioactive iodine treatment, DTC is still a stubborn and curable disease in most patients, while the cure rate of MTC is low, depending on early diagnosis. Most ATCs are incurable. In recent years, great progress has been made in identifying genetic changes in thyroid cancer. Genetic testing of FNA samples or blood samples provides useful information for clinical decision-making. Tumor staging, whether after surgery or through imaging examinations, as well as measurement of tumor markers thyroglobulin (DTC) and calcitonin (MTC), can be used for dynamic risk stratification for subsequent surgery [5]. In advanced metastatic thyroid cancer, the use of tyrosine kinase receptor inhibitors (including sorafenib, lenvatinib, vandetanib, and cabozantinib) for molecular targeted therapy can help control tumor progression and prolong progression-free survival. Using dynamic risk stratification methods to manage thyroid cancer, compared with other cancers, the treatment effect of most patients with thyroid cancer is excellent. The main challenge in the future is to identify high-risk patients and to treat and monitor them appropriately [6]. However, he did not propose how to identify high-risk patients and propose appropriate treatment and detection methods. In order to prepare ligand-modified microbubbles for targeted ultrasound imaging, it is important to maximize the amount of the ligand associated with the bubble shell. Unnikrishnan et al. described the optimization of the use of biocompatible cosurfactants in the microbubble formulation medium to maximize the incorporation of the targeting ligand-lipid conjugate into the microbubble shell [7], thereby reducing the amount of amalgam preparation and the ligand ratio of microbubbles to independent bubbles [8]. The effect of the concentration of the cosurfactant propylene glycol (PG) on the efficiency of preparing microbubbles by amalgamation and the degree of association between the fluorescent PEG-lipid and the microbubble shell was tested. Then, three sets of targeting bubbles, VCAM-1-targeting peptide VHPKQHRGGSK (FITC) GC-PEG-DSPE, cyclic RGDfK-PEG-DSPE, and right *α*_*Vβ*_3__ and control cRADfK-PEG-DSPE without this affinity were prepared. Microbubbles were prepared by 45 s combination, with DSPC and PEG stearate as the main components. However, Bychkov's experiment needs more data to support, especially whether the contrast agent can be used well under any circumstances [9]. The Tian virtual reality visual display system creates a real virtual product display system that allows users to swim and perform interactive operations in a three-dimensional virtual environment, thereby completely simulating the shopping selection and payment process in reality so that users have an immersive experience. It aims to realize the design of the immersive 5G virtual reality visual display system through big-data digital city technology [10]. Using the big-data digital city technology, an immersive virtual reality visualization system is designed and implemented from the visual, auditory, and tactile three-dimensional display modes [5], providing users with a real and interactive three-dimensional visualization environment and enabling users to have more intuitive vision experience. The experimental results show that the smoothness of the virtual reality visualization system test can reach 60 FPS, the good rate is nearly 33%, and the good rate of realistic feedback of the model scene is about 62.5%. However, the virtual reality visual display system has not yet been widely used because of the lack of extensive testing and high cost [11].

RETRACTED

The innovations of this article are as follows: (1) combining theory with practice, fully applying theoretical foundations in practice, and discussing the application of virtual reality technology combined with contrast-enhanced ultrasound in the diagnosis and treatment of thyroid cancer; (2) combining qualitative with quantitative. The combination of research includes both data analysis and qualitative content analysis.

## 2. The Clinical Research Method of Virtual Reality Augmented Technology Combined with Contrast-Enhanced Ultrasound in the Assessment of Thyroid Cancer

### 2.1. Thyroid Cancer

#### 2.1.1. Understanding of Thyroid Cancer

Among the malignant tumors of the endocrine system, thyroid cancer is the most common, accounting for about 96.2%. In recent years, the global incidence of thyroid cancer has continued to rise, and the incidence of female malignant tumors in my country has reached the fifth place in the world [12]. And the incidence rate is higher in coastal areas and cities. Although most thyroid cancers have a good prognosis, according to data, the 5-year survival rate of thyroid cancer patients in the United States is as high as 98.1%, while these data in my country are only 84.3% [13]. In addition, up to 20% of patients with thyroid tumors are already at a high-risk stage when they are first diagnosed.

#### 2.1.2. Causes of Thyroid Cancer

The increase in the incidence of thyroid cancer is related to the patient's age, gender, weight, family history, and other factors. This study shows that about 43% of patients with thyroid cancer are 45–64 years old [14]. Overweight and obesity are independent risk factors. With the increase in the incidence of thyroid cancer, there are more and more studies on its etiology and pathogenesis [15].

The relationship between iodine intake and thyroid cancer is currently unclear. Most scholars believe that excessive iodine intake is a risk factor for thyroid cancer [16]. A few scholars believe that high iodine can reduce the risk of thyroid cancer. High iodine can inhibit the proliferation of cancer cells and promote the apoptosis and migration of cancer cells. It is a protective factor for thyroid cancer [17]. Past animal experiments have shown that iodine deficiency will increase the incidence of thyroid cancer. Studies have found that iodine deficiency can cause abnormal proliferation of thyroid cells and increase their sensitivity to ionizing radiation. In addition, when acting as an antioxidant, iodine deficiency may increase the oxidative burden of cells [18], thereby increasing DNA damage and chance of mutation. Another scholar found that, in areas with sufficient iodine, patients with thyroid nodules with relatively low iodine intake have a higher risk of cancer than patients with relatively average iodine intake [19]. However, there is no more research to support the relationship between relatively low iodine intake and the risk of thyroid cancer. Thyroid glands are particularly sensitive to the long-term effects of radiation exposure, and studies on humans exposed to sublethal radiation doses have proved this view. Damage from radiation exposure may lead to cell apoptosis, cell cycle arrest, DNA repair, and cancer.

RETRACTED

#### 2.1.3. Pathogenesis of Thyroid Cancer

Thyroid tumors are derived from two different cell groups, parafollicular cells and follicular cells, which are basically divided into differentiated carcinomas, poorly differentiated carcinomas, and undifferentiated carcinomas [20]. Thyroid cancer differentiated from cells, accounting for about 90%, is basically divided into papillary or follicular shape. The most common histological type is papillary thyroid carcinoma, which is more responsive to treatment and usually has a good prognosis [21]. On the contrary, poorly differentiated and undifferentiated thyroid cancer is more aggressive and lethal, but fortunately, its prevalence is lower than differentiated thyroid cancer [22].

Regarding the process of tumor formation and its heterogeneity, there are currently two main hypotheses: a classic (random) multistep carcinogenesis model based on the theory of tumor clonal origin and the latest hypothesis based on cancer stem cells [23]. Multistep models show that the formation of tumors is the result of genome instability in somatic cells and is the emergence of more aggressive clones that can survive under the pressure of microenvironment selection [24]. The emergence of functionally significant mutations leads to the differentiation of new subclones, which can control and compete with other cells, leading to homogenous tumors, until new, important, and more comprehensive mutations appear [25]. According to this theory, thyroid follicular carcinoma is believed to originate from follicular epithelial cells.

The second hypothesis is the thyroid cancer stem cell model, which assumes that, after genetic and epigenetic transformation, there is a small subset of stem cells that may produce cancer cells with different phenotypes [26]. Some models point out that, after genetic changes, thyroid stem cells will produce untransformed thyroid stem cells, and untransformed thyroid stem cells will produce a type of pluripotent progenitor cell called thyroid blast, which is easy to develop into PTC, and benign tumors are formed by thyroid precursor cells (primary cells) [27]. Activation of this pathway stimulates cell proliferation, and activation of its components promotes tumorigenesis [28].

RETRACTED

#### 2.1.4. Preoperative Diagnosis of Thyroid Cancer

Thyroid function testing, ultrasonography, and fine-needle aspiration are the cornerstones of the preoperative diagnosis and evaluation of thyroid cancer. Other examination methods such as neck CT, PET-CT, and thyroid cancer functional metabolism imaging also have certain value in the preoperative diagnosis of thyroid cancer [29]. The value of the thyroid hormone is increasingly recognized because of its ability to promote the proliferation of thyroid tumors. In vitro experiments have found that A indicates that the thyroid hormone has the effects of stimulating tumor growth and antiapoptosis in thyroid diseases [30]. Another clinical study found that patients with hyperthyroidism have a higher risk of thyroid cancer. The longer the duration of hyperthyroidism, the higher the risk of thyroid cancer. Regarding the determination of the level of the thyroid-stimulating hormone, there are different opinions on the risk of thyroid cancer [31]. The data show that the serum concentration of TSH is an independent predictor for the diagnosis of malignant thyroid tumors. Patients with aggressive thyroid cancer have higher preoperative serum TSH concentrations, suggesting that TSH has a potential role in the progression of differentiated thyroid cancer. A prospective study found that the increased risk of thyroid cancer was associated with lower TSH7K levels (<0.5 mU/l) [32]. Ultrasonography has become the first choice for clinicians to screen and evaluate the nature of thyroid nodules because of its real-time, dynamic, low-cost, noninvasive, and simple advantages. Conventional grayscale ultrasound examination of the thyroid gland indirectly evaluates the benign and malignant nodules through the echo, texture, margin, calcification, and morphology of the nodules. However, the single ultrasound feature cannot balance sensitivity and specificity to more than 85% when diagnosing thyroid cancer [4]. Therefore, the research of virtual reality augmented technology combined with ultrasound features has practical significance and is of great value for clinical research [33].

#### 2.1.5. Pathological Classification of Thyroid Cancer

Differentiated thyroid cancer (DTC) is the most common thyroid cancer, accounting for more than 95% of the total [34]. Poorly differentiated thyroid cancer (PDTC) is a kind of follicular-derived TC that is more aggressive than DTC. DTC includes papillary thyroid carcinoma (PTC), as shown in Figures 1(c)–1(f), and follicular thyroid carcinoma (FTC), as shown in Figures 1(a) and 1(b). PTC is the most common, with good prognosis, easily metastasizes to cervical lymph nodes, and has less metastasis to the lung. FTC, Hurthle cell carcinoma, and PDTC are less common, but the risk is higher, and it is easy to metastasize to distant parts, especially the lungs and bones. Anaplastic thyroid cancer (ATC) is extremely rare (<1%). The tumor progresses rapidly. Patients often experience dumbness and difficulty in swallowing and breathing, and most of them appear as large, hard goiter masses with or without lymph node metastasis (LNM). Once ATC is found, a rapid biopsy should be given, and the systemic metastasis should be assessed at the same time. ATC often occurs at the same time as DTC. Therefore, clinicians should pay close attention to whether the above symptoms occur in DTC patients with a long history. Due to its rapid growth and poor prognosis, possible treatments are still in clinical trials and are expected to improve the prognosis of ATC [35]. Medullary thyroid cancer (MTC) accounts for only 1% of all TCs and has neuroendocrine function [36]. The common age of onset is 40–60 years. The disease has a high incidence of cervical LNM. About 70% of MTC patients have LNM during surgery, and cervical lymph node lesions are mostly the first symptom.  Figure 1 shows the pathological classification of thyroid cancer.

RETRACTED

### 2.2. Contrast-Enhanced Ultrasound

Contrast-enhanced ultrasound (CEUS) uses local intravenous injection of the contrast agent SonoVue. Due to changes in the volume of the contrast microbubbles due to the effect of sound pressure, the gas-liquid connection will generate strong sound signals and harmonic signals, which may generate strong noise. In order to enhance the Doppler blood flow signal, CEUS diagnoses the disease by observing the microvascular distribution of the tissue structure and can evaluate the noninterventional hemorrhage of the bleeding organs. SonoVue is a true blood concentration contrast agent, widely used in abdominal organs such as the liver and kidney. The role of contrast ultrasound in the diagnosis of liver diseases is described in the instructions. Ultrasound technology to improve contrast is a hot spot in medical ultrasound research, which can provide the characteristics of OECD small blood vessel hemorrhage. Since the current ultrasound contrast agent requires a low resonance frequency, its application in thyroid diseases is still in the active exploration and application stage.

Ultrasound elastography (US-E) has received wide attention from clinicians since it was proposed by Ophir in 1991. US-E was proposed to be used to distinguish between thyroid cancer and benign nodules. Assessed by hardness, malignant lesions are often stiffer than normal tissues. US-E artificially exerts an external force on the tissue to transform the signal amplitude changes before and after compression into color images. However, this new technology is not highly accepted. When determining the level of flexibility, the classification may be subject to a certain degree of subjective influence. In order to reduce the variability, the research is based on more significant numerical score classification, which is too time-consuming for objective analysis. Therefore, ultrasound elastography may be a promising tool for the assessment of thyroid nodules, but it has not been routinely implemented.

RETRACTED

### 2.3. Virtual Reality Augmented Technology

Although the indications for the widely used fine-needle aspiration (FNA) have been clear, there are still false negatives. These false negatives not only reduce the accuracy of diagnosis but also produce many unnecessary invasive tests. On the contrary, the increasing demand for diagnosis also brings difficulties to the implementation of standards, data analysis, and processing; therefore, there is an urgent need for a better method. At the beginning of the twenty-first century, virtual reality technology, a branch of computer science, provides a new development direction for medical imaging. Based on the integration of multidisciplinary big data, an efficient intelligent diagnosis system will help the promotion of thyroid ultrasound diagnostic standards in the future.

Traditional ultrasound has its limitations. It cannot distinguish certain diseases such as adenoma and nodular goiter. The diagnosis result depends more on the sonographer, and the subjectivity is strong, which leads to differences between doctors at different diagnostic levels. In addition, with the increase in the number of patients and the increase in scanning time, the burden of thyroid ultrasound scanning physicians has also increased. Virtual reality augmented technology can make up for the inevitable limitations of traditional ultrasound and compare the diagnostic criteria of thyroid nodules with the enhancement technology. Combined, it can significantly improve the diagnosis of thyroid.

In summary, the combination of contrast-enhanced ultrasound and virtual reality augmented technology, as a new differential diagnosis technology for thyroid cancer, provides a new diagnostic method and exerts its inherent advantages. Virtual reality augmented technology combined with contrast-enhanced ultrasound will further improve the accuracy of thyroid cancer diagnosis, and it is worthy of further research. The application of virtual reality augmented technology in the ultrasound diagnosis of thyroid cancer will greatly improve the diagnostic value, stability, and efficiency and has broad application prospects.

RETRACTED

### 2.4. Fuzzy Clustering Algorithm

#### 2.4.1. Fuzzy Mean Clustering Algorithm

FCM is a fuzzy combination method proposed by Bezdek, which is widely used in segmentation and image recognition. FCM is a fuzzy combination based on the image space and is basically a nonlinear iterative optimization method based on target operations. If the image pixel is composed of *n* sample sets, *X* = {*x*_*i*_|1, 2,…, *n*}, then the image segmentation problem is transformed into the problem of dividing these *n* samples into *c* categories. Target FCM algorithm is repeated by selecting the appropriate fuzzy membership and focus, and the operation target is suppressed to a minimum, for the maximum segmentation effect. The objective function of FCM is

(1) $$\begin{array}{c} H_{\text{FCM}}=\sum_{m=1}^{t}\sum_{n=1}^{u}\varsigma_{mn}^{i}{\left\|x_{n}-y_{m}\right\|}^{2}. \end{array}$$

Among them, *i* is the fuzzy index, which controls the fuzzy degree of the clustering result. In general, *i* = 2. *y*_*m*_ represents the cluster center point, the probability that the *m*th pixel *ς*_*mn*_ belongs to the *n*th cluster center point, and ‖•‖ represents the Euclidean distance. According to the Lagrangian conditional extreme value method, the necessary conditions for the objective function *H*_FCM_ to take the minimum value are obtained:

(2) $$\begin{array}{c} \varsigma_{mn}=\frac{{\left[1/{\left\|x_{n}-y_{m}\right\|}^{2}\right]}^{1/i-1}}{\sum_{k=1}^{c}{\left[1/{\left\|x_{n}-y_{k}\right\|}^{2}\right]}^{1/i-1}}, \end{array}$$

(3) $$\begin{array}{c} y_{m}=\frac{\sum_{i=1}^{n}\varsigma_{mn}^{i}x_{m}}{\sum_{i=1}^{n}\varsigma_{mn}^{i}}. \end{array}$$

In the process of image segmentation, the traditional FCM algorithm only considers the gray-level histogram information of the image and fails to consider the gray-level correlation between each pixel and its neighboring pixels, which makes the algorithm very sensitive to noise. In order to improve the antinoise performance of the FCM algorithm, researchers have proposed many improved methods of FCM, including the FCM segmentation method based on the space constraint condition of the distance measurement kernel and the image segmentation algorithm that extracts the 5-dimensional neighborhood features of pixels and performs progressive clustering. Although the improved methods have their own merits, the neighborhood constraint introduces one or more neighborhood constraints into the objective function of the FCM to form a penalty term, taking the objective correlation between image pixels into consideration. Among them, the most classic is to use the neighboring pixels around each pixel as a constraint condition to join the FCM objective function:

(4) $$\begin{array}{c} H_{\text{FCM}-\text{s}}=\sum_{m=1}^{t}{\sum_{n=1}^{u}\varsigma_{mn}^{i}\left\|x_{n}-y_{m}\right\|}^{2}+\frac{\beta }{P_{R}}\sum_{m=1}^{t}\sum_{n=1}^{u}\varsigma_{mn}^{i}\left(\underset{x_{r}\in N_{i}}{\sum }{\left\|x_{r}-y_{n}\right\|}^{2}\right). \end{array}$$

*N*_*i*_ is a neighborhood pixel with pixel *x*_*i*_ as the center, and *P*_*R*_ is the rank of *N*_*i*_. *x*_*r*_ is the gray value of the neighboring pixels around pixel *x*_*i*_. Due to the complexity of the neighborhood term and the long calculation time, some researchers proposed to replace the neighborhood term with the mean or median value in the neighborhood window; then, the objective function (equation (4)) is changed to

(5) $$\begin{array}{c} H_{\text{FCM}-\text{sl}}=\sum_{m=1}^{t}\sum_{n=1}^{u}\varsigma_{mn}^{i}{\left\|x_{n}-y_{m}\right\|}^{2}+\beta \sum_{m=1}^{t}\sum_{n=1}^{u}\varsigma_{mn}^{i}{\left\|{\bar{x}}_{n}-y_{m}\right\|}^{2}, \end{array}$$

where ${\bar{x}}_{n}$ represents the median or mean value of neighboring pixels.

RETRACTED

#### 2.4.2. Multiscale Fuzzy C-Means Clustering

The main idea of MsFCM is to use the anisotropic diffusion (AD) filtering method to construct a set of multiscale images from coarse to fine, gradually on the multiscale images, calculate the membership value of each pixel in the image, and divide and classify each point according to the membership value to achieve image segmentation.

(6) $$\begin{array}{c} \text{MsFCM}=\sum_{m=1}^{t}\sum_{n=1}^{u}\tau_{mn}^{i}{\left\|x_{m}-y_{n}\right\|}^{2}+\frac{\phi }{P_{R}}\sum_{m=1}^{t}\sum_{n=1}^{u}\tau_{mn}^{i}\sum_{r\in N_{i}}{\left\|x_{r}-y_{n}\right\|}^{2}+\delta \sum_{m=1}^{t}\sum_{n=1}^{u}{\left(\tau_{mn}-\tau_{mn}^{\prime }\right)}^{i}{\left\|x_{m}-y_{n}\right\|}^{2}. \end{array}$$

The sum *φ*_*δ*_ is the weighting coefficient, in which *τ*_*mn*_ represents the membership value of the pixel at the current scale, and *τ*_*mn*_′ is the membership value of the previous scale. The objective function contains three terms. The first item is the objective function of the traditional FCM. The pixel points are classified into the category closest to the center point through the judgment of the membership value. The second item is to consider the spatial information of the image and adjust the cluster center point through the membership degree of the neighboring pixels. In the third item, the pixel membership value of the previous scale is used as the supervision item to adjust the membership value of the current scale to fully consider the information between the front and back scales. Here, *τ*_*mn*_′ is obtained by comparing the membership value of the previous scale pixel with the threshold *k* (in this article, it is set to 0.85), and the relationship is

(7) $$\begin{array}{c} \tau_{mn}^{\prime }=\left\{\begin{array}{c} \tau_{mn}^{\prime }\text{ if}\max\left(\tau_{mn}^{\prime }\right)>k,\\ 0,\text{others}. \end{array}\right. \end{array}$$

RETRACTED

#### 2.4.3. Multiscale Image Construction Based on SRAD Filtering

For the speckle noise in the ultrasound image, some researchers use the speckle reducing anisotropic diffusion (SRAD) filtering method to filter out. SRAD performs iterative filtering based on the following partial differential equations:

(8) $$\begin{array}{c} \left\{\begin{array}{c} \frac{\partial \left(m,n,t\right)}{\partial t}=\text{div}\left[w\left(q\right)\nabla L\left(m,n,t\right)\right],\\ L\left(m,n,0\right)=L_{0}\left(m,n\right). \end{array}\right. \end{array}$$

In the formula, a grayscale image *L*_0_(*x*, *y*) is given. The image *L*(*m*, *n*, *t*) after denoising with time *t* is *L*(*m*, *n*, *t*), *w*(*q*) is the diffusion coefficient, *q* is called the instantaneous change operator and is the edge detector in SARD, and *t* represents the diffusion time. In this paper, it is set as a discrete number, *t*=*u* · *n*_*t*_ · Δ*t*, in which *u*=1,2,…, *U* is the scale, *u∗n*_*t*_ is the number of iterations, and *n*_*t*_ is set as the iteration interval Δ*t* to represent the time step. When *u* = 1, it is the finest image scale, and when *u* = *U*, it is the roughest image scale.

#### 2.4.4. Simplification of Field Items

This paper adopts the idea of improving formula (4) into formula (5), simplifies the traditional MsFCM algorithm (equation (6)), and replaces the domain term in the formula with the median *i*_*x*_ of the neighborhood pixel. The objective function of MsFCM after simplification is

(9) $$\begin{array}{c} {\text{MsFCM}}_{M}=\sum_{m=1}^{t}\sum_{n=1}^{u}\tau_{mn}^{i}{\left\|x_{m}-y_{n}\right\|}^{2}+\varphi \sum_{m=1}^{t}\sum_{n=1}^{u}\tau_{mn}^{i}{\left\|{\bar{x}}_{m}-y_{n}\right\|}^{2}+\delta \sum_{m=1}^{t}\sum_{n=1}^{u}{\left(\tau_{mn}-\tau_{mn}^{\prime }\right)}^{i}{\left\|x_{m}-y_{n}\right\|}^{2}. \end{array}$$

After simplification, the algorithm is more efficient and practical.

#### 2.4.5. Particle Swarm Optimization Algorithm

The particle swarm optimization algorithm completes global optimization by tracking the best solution detected by each particle and the overall best solution of the particle swarm. Suppose that the initial value of the particle swarm optimization algorithm is a random particle group, and each particle has its own position and velocity. The extreme value and global extreme value of each particle are dynamically monitored to update the position and velocity. They satisfy the following relationship:

(10) $$\begin{array}{c} \left\{\begin{array}{c} p_{i,j}^{o+1}=p_{i,j}^{o}+t_{1}\cdot {\text{rand}}_{1}\left(\;\right)\cdot \left(j{\text{best}}_{i,j}^{o}-q_{i,j}^{o}\right)+t_{2}\cdot {\text{rand}}_{2}\left(\;\right)\cdot \left(g{\text{best}}_{i}^{o}-q_{i,j}^{o}\right),\\ q_{i,j}^{o+1}=q_{i,j}^{o}+p_{i,j}^{o}. \end{array}\right. \end{array}$$

Usually, a value of 2 is set for both *t*_1_ and *t*_2_. rand_1_()() and rand_2_()() are random numbers between 0 and 1, in which *j*best_*i*,*j*_ are the optimal extreme points of individual particles and *g*best_*i*,*j*_ are the optimal extreme points of all particles.

RETRACTED

The individual particle extreme point (*j*best) and the global extreme point (*g* best) of the population are determined by the fitness function value in the PSO. The fitness function here is the objective function of the MsFCM algorithm (equation (9)), and the particle position corresponds to the cluster center point; the dimension of the particle represents the number of clustering classes; then, the fitness function of PSO is

(11) $$\begin{array}{c} l\left(j\right)=\sum_{m=1}^{t}\sum_{n=1}^{u}\tau_{mn}^{i}{\left\|x_{m}-y_{i,j}\right\|}^{2}+\phi \sum_{m=1}^{t}\sum_{n=1}^{u}\tau_{mn}^{i}{\left\|{\bar{x}}_{m}-y_{i,j}\right\|}^{2}+\delta \sum_{m=1}^{t}\sum_{n=1}^{u}{\left(\tau_{mn}-\tau_{mn}^{\prime }\right)}^{i}{\left\|x_{m}-y_{i,j}\right\|}^{2}. \end{array}$$

According to the constraints of each pixel ∑_*j*=1_^*c*^*τ*_*ij*_=1, the Lagrangian method is used to solve the membership value of each pixel:

(12) $$\begin{array}{c} \tau_{mn}=\frac{1+\delta \sum_{k=1}^{c}\tau_{mk}^{\prime }{\left\|x_{m}-y_{i,j}\right\|}^{2}-\tau_{nk}^{\prime }{\left\|x_{m}-y_{k,j}\right\|}^{2}/\left(1+\delta \right){\left\|x_{m}-y_{k,j}\right\|}^{2}+\phi {\left\|{\bar{x}}_{m}-y_{k,j}\right\|}^{2}}{\sum_{k=1}^{c}\left(1+\delta \right){\left\|x_{m}-y_{i,j}\right\|}^{2}+\phi {\left\|{\bar{x}}_{m}-y_{i,j}\right\|}^{2}/\left(1+\delta \right){\left\|x_{m}-y_{k,j}\right\|}^{2}+\phi {\left\|{\bar{x}}_{m}-y_{k,j}\right\|}^{2}}. \end{array}$$

Each particle is updated iteratively according to equations (10) and (11) until the specified number of iterations or the specified error standard is met. At this time, the global extremum *g* best is the global optimal clustering center point, so an optimal global clustering center point can be found on each scale image and then used to segment the CEUS image.

RETRACTED

In order to objectively evaluate the segmentation results, this paper uses segmentation accuracy (SA) and edge retention (Pratt's figure of merit, FOM) to measure the segmentation results of these four clustering methods. SA represents the overlap rate between the real result and the segmentation result, and the function expression is

(13) $$\begin{array}{c} \text{SA}=\frac{Y_{\text{correct}}}{Y_{\text{total}}}. \end{array}$$

*Y*_correct_ is the number of pixels correctly classified, and *Y*_total_ represents the total number of pixels in the image. FOM is a parameter that characterizes the performance of image edge retention, and its expression is as follows:

(14) $$\begin{array}{c} \text{FOM}=\frac{1}{\max\left\{Y_{1},Y_{R}\right\}}\sum_{i=1}^{N_{R}}\frac{1}{1+d_{i}^{2}\alpha }. \end{array}$$

FOM is related to the method of edge detection. This paper uses Canny edge detection. The value range of FOM is [0, 1]; the closer the value is to 1, the closer the boundary of the segmentation result is to the real contour.

(15) $$\begin{array}{c} E=\int_{0}^{1}\left[\frac{1}{2}\left(\alpha \left(s\right){\left|U{}^{\prime }\left(s\right)\right|}^{2}+\beta \left(s\right){\left|U{}^{\prime \prime }\left(s\right)\right|}^{2}+E_{\text{ext}}\left(U\left(s\right)\right)\right)\right]\text{d}s. \end{array}$$

The above formula represents the energy function definition formula of snakes; *E*_ext_ represents the external energy of the image, which is generally defined as the energy generated by the gradient field of the image.

## 3. Clinical Research Experiment of Virtual Reality Augmented Technology Combined with Contrast-Enhanced Ultrasound in Evaluating Thyroid Cancer

### 3.1. Subjects of Clinical Research on Thyroid Cancer

This article selected 2104 cases of thyroid surgery performed in Y Hospital from 2018 to 2019, of which 359 cases (75.6%) were pathologically diagnosed as TC. A total of 91 cases (5.7%) were excluded, among which 90 cases (5.6%) had secondary operations, 5 cases (0.03%) had incomplete information, and 7 cases (0.04%) had other types of malignant tumors. In the end, the study included a total of 258 TC patients with complete information after the first operation.  Table 1 is a comparison of the general data of benign and malignant thyroid nodules.

1. Inclusion criteria: those who were confirmed to be TC by histopathological report
2. Exclusion criteria: out-of-hospital surgery patients; recurrent TC or a history of TC; nonprimary TC and parathyroid disease; incomplete information

The identification variables of all participants are deleted, and anonymous data are used to ensure privacy and confidentiality. Only investigators have access to these data. All procedures performed in the research are in compliance with the ethical standards of the Institutional Research Committee and in compliance with the 1964 Declaration of Helsinki and its subsequent amendments or similar ethical standards.

RETRACTED

### 3.2. Research Methods

#### 3.2.1. Instrument and Contrast Agent

The instrument and contrast agent are as follows: Philips EPIQ 7 ultrasonic diagnostic apparatus (Philips Medical Corporation, Germany), probe 12L-5 (frequency: 5.0–10.0 MHz), SonoVue (Bracco SpA, Milan, Italy) as the contrast agent, and the venous access established by the elbow vein. 25 mg of the contrast agent is dissolved in 5 ml of 0.9% sodium chloride and shaken repeatedly to prepare microbubble suspension. The patient takes the supine position, the neck is fully stretched, and the front area of the neck is exposed. First, routine ultrasound is used to examine the thyroid nodules to determine their morphology, boundary, and internal echo characteristics. Then, color Doppler ultrasound is used to examine the thyroid nodules and surrounding tissues to determine the blood flow in and around the lesion. Combined with the results of conventional ultrasound and color Doppler ultrasound, the best observation section of the thyroid nodule was determined. Then, the probe was fixed, and the contrast pulse sequence of the instrument was turned on. Then, 2.4 ml of the prepared SonoVue contrast medium microbubble suspension was quickly injected into the blood vessel through the cubital vein, and then 5.0 ml of normal saline was injected immediately. Data were collected when the contrast agent was injected. Continuous real-time dynamic observation of the detection area and full video recording under the low mechanical index and double-frame imaging mode were done. If the obtained thyroid nodule contrast image is unsatisfactory, the contrast agent is reinjected through the cubital vein for a second ultrasound contrast.

### 3.3. Observation Indicators

(1) The components are specifically divided into solid, mixed (including cystic-based and solid-based), and cystic; (2) echo specifically refers to extremely low echo, low echo, and equal/high echo; (3) edge is divided into regular and irregular; (4) calcification is divided into spot-like strong echo, coarse calcification, and no strong echo; (5) shape is divided into aspect ratio >1 and aspect ratio <1. Diagnostic power: sensitivity, specificity, positive predictive value (PPV) and negative predictive value (NPV), and accuracy.

### 3.4. Image Analysis Method

The ultrasound report and image data of the included thyroid nodules are strictly trained by me, and the images are standardized with reference to the thyroid ultrasound description dictionary. Before viewing the pathological results, the ultrasound performance of the thyroid tumor is analyzed and recorded. For signs of doubt, please consult with the instructor for agreement; for multicenter nodules, code and record separately according to the location and size of the nodules. The main record content is as follows:

1. Ingredients: cystic (almost all cystic), cystic-solid (the cystic and solid parts are mixed in a similar proportion), sponge-like (multiple small anechoic structures can be seen inside the nodule, and the volume of these anechoic structures has exceeded half of the total volume of the nodules, and solidity (almost all solidity).
2. Echo level: referring to the thyroid parenchymal echo and anterior neck muscle group echo, it is divided into very low echo, hypoechoic, isoechoic, hyperechoic, mixed echo, and anechoic. Very hypoechoic is the echo below the anterior cervical muscle layer; hypoechoic is the echo lower than the thyroid parenchyma itself, but higher than the echo of the anterior cervical muscle layer; isoecho is equivalent to the echo of the thyroid parenchyma; hyperechoic is higher than the thyroid gland substantial echo. When the proportion of solid components in a cystic-solid nodule is higher than 80%, the echo level of the solid component shall be recorded as the standard; when the echo level of the solid nodule is different, the echo level of the dominant part is recorded.
3. Aspect ratio: the measured values of the longitudinal and transverse diameters are taken when the thyroid cross section is selected, and the ratio of the longitudinal diameter to the transverse diameter is calculated, which is divided into <1 and ≥1.
4. Boundary: it is divided into clear and unclear; clear means that the thyroid nodule can be clearly separated from the surrounding thyroid parenchyma, and unclear means that there is no clear boundary between the thyroid nodule and the surrounding thyroid parenchyma, and the two cannot be separated.
5. Morphology: it is divided into regular and irregular. Regular shapes include regular circles and ellipses. Irregular shapes include leaf-like, burr-like, or angular protrusions.
6. Envelope invasion: the nodule involves or breaks through the thyroid capsule, which is divided into presence and absence. Special attention should be paid when the nodule causes the bulge of the capsule.
7. Calcification: it is divided into microcalcification, gross calcification, marginal calcification, and comet tail sign. Microcalcifications are spot-like strong echoes with a diameter of <1 mm; coarse calcifications are strong echoes with a diameter of ≥1 mm. They are divided into clumps, bands, arc-shaped, and edge calcifications according to their appearance and shape. According to whether there is a comet tail sign behind the calcification, it is marked whether the nodule is accompanied by a comet tail sign; if there is no calcification, it means that there is no calcification in the nodule.

RETRACTED

### 3.5. Statistical Processing

The statistical analysis in this paper adopts the SPSS 19.0 version and uses the arithmetic mean, standard deviation (SD), median, and other methods to summarize continuous variables; the categorical variables were divided by weighted frequency and percentage (%). Continuous variables were analyzed by the *t*-test, and categorical variables were analyzed by the chi-square test; *P* < 0.05 indicated that the difference was statistically significant. In addition, the selection bias was reduced by including all TC patients. Considering that this study is a retrospective study, the directional bias cannot be ruled out.

## 4. Clinical Research Analysis of Virtual Reality Augmented Technology Combined with Contrast-Enhanced Ultrasound in the Assessment of Thyroid Cancer

### 4.1. Comparison of Contrast-Enhanced Ultrasound Signs

As can be seen from Table 2 and Figure 2, the results of ultrasound signs in the identification of benign and malignant thyroid nodules are quite different. For example, in the aspect ratio, the proportion of benign aspect ratio <1 reached 94.3%, the proportion of malignant aspect ratio ≥1 reached 58.3%, the good proportion of benign nodules was 93.2%, and the envelope of malignant nodules was invaded, accounted for 34.2%. In addition, the benign and malignant nodules in the above items are comparable and statistically different (*P* < 0.05).

### 4.2. Ultrasound Contrast Enhancement Results

The method of nodular contrast enhancement in this group is shown in Table 3 and Figure 3. In 18 cases of nodular goiter, there were 3 cases of low enhancement, 5 cases of equal enhancement, 9 cases of high enhancement, and 5 cases of uneven enhancement; most of them were benign nodules which showed equal enhancement and high enhancement; 12 cases of malignant nodules showed low enhancement, 6 cases showed high enhancement, and 5 cases showed uneven enhancement.

The results of contrast-enhanced ultrasound and pathology are shown in Table 4 and Figure 4. The *P* values of the items grouped in this article are all less than 0.05, which is statistically significant. The number of uneven angiographic images of malignant nodules was relatively large, 36 cases, which was much higher than the number of uneven cases in benign nodules, 27 cases. Malignant pathology showed unclear boundaries, accounting for more than 50%, while benign pathology was only 15 cases, accounting for 22.3%. The time of malignant pathological perfusion is also slow, while the time of benign pathological perfusion is synchronous.

RETRACTED

### 4.3. Multivariate Logistic Analysis Results and Risk Factor Assessment of Thyroid Cancer

Using the TI-RADS classification and description method, thyroid nodules were evaluated by physicians of different years. The results are shown in Table 5 and Figure 5. From the perspective of the *K* value, we can see that the value of microcalcification is 0.784, the value of aspect ratio ≥1 is 0.787, and the value of internal blood flow is 0.683, indicating that the three indicators are in good agreement; and the solid *K* value is only 0.264, indicating that its consistency is very weak.

Taking pathological results as the dependent variable and suspicious independent risk factors of thyroid cancer as the independent variable, a multivariate logistic regression analysis was performed. The regression results are shown in Table 6 and Figure 6. Suspicious independent risk factors for thyroid cancer, according to the OR value, are in the order of microcalcification, irregular shape, very low echo, aspect ratio ≥1, low echo, unclear border, and solid nodules. One point is assigned to the smallest partial regression coefficient *β* value of 0.969, the ratio of the partial regression coefficient *β* value of other signs to 0.969 is assigned to each sign, and 10 times the value of each sign is assigned as the final weight score of the sign to construct thyroid cancer. The risk assessment scale was again included in the logistic regression analysis, and the total score of each nodule was used to establish a thyroid cancer diagnostic model.

### 4.4. Diagnostic Efficacy of Ultrasound Signs

It can be seen from Table 7 and Figure 7 that, among the 8 signs of malignant thyroid nodules, the most sensitive is solid, followed by hypoechoic; the higher specificity is followed by capsule invasion, aspect ratio ≥1, and distant field echo attenuation; the order of higher accuracy is aspect ratio ≥1, membrane invasion, far-field echo attenuation, irregular shape, and microcalcification; the order of larger ratio is aspect ratio ≥1, solidity, far-field echo attenuation, irregular shape, and microcalcification; positive likelihood ratio >10 is aspect ratio ≥1.

Table 8 and Figure 8 show the results of different diagnostic cutoff points classified by virtual reality technology and CEUS in the joint diagnosis of risk. Judging from different diagnostic cutoff points, the accuracy of combined diagnosis is higher, and the sensitivity value is higher. When the diagnostic cutoff points are 14.2 and 19.3, the sensitivity is the highest at 0.954. Although the diagnostic cutoff points are constantly changing, their sensitivity exceeds 85%. When using contrast-enhanced ultrasound to diagnose thyroid nodules, the sensitivity and specificity values should be selected. High is the best cutoff point.

RETRACTED

## 5. Conclusion

This article mainly focuses on the clinical research of virtual reality augmented technology combined with contrast-enhanced ultrasound in the assessment of thyroid cancer. It uses literature methods and experimental research methods to design a clinical experiment of virtual reality augmented technology combined with contrast-enhanced ultrasound in the assessment of thyroid cancer and analyzes contrast-enhanced ultrasound signs' comparison and diagnostic efficiency. The diagnostic sensitivity and specificity of virtual reality augmented technology combined with contrast-enhanced ultrasound for thyroid cancer exceed 85%, which is a major breakthrough in the development of ultrasound imaging technology. There are many shortcomings in this study. The sample size is small, and it is not a multicenter study. Part of the pathological results of the study of malignant signs of thyroid nodules lacks the basis for the identification of thyroid follicular tumors. This study did not group the size of thyroid nodules in detail. Research and the evaluation of nodule elastography and contrast-enhanced ultrasound may have ultrasound differences caused by different sizes. In summary, we still need to further increase the sample size and continue in-depth research in the future. We believe that, with the development of ultrasound contrast technology and virtual reality technology, through the continuous discovery of a new generation of ultrasound contrast agents, we will further explore more penetrating and stable contrast agents to improve the diagnosis of more diseases.

## Figures and Tables

**Figure 1:** Pathological classification of thyroid cancer.

**Figure 2:** Comparison of different ultrasound signs in differentiating benign and malignant nodules.

**Figure 3:** Contrast enhancement mode of thyroid nodules.

**Figure 4:** CEUS enhancement mode and pathological comparison results.

**Figure 5:** Consistency results of TI-RADS descriptors for physicians of different years.

**Figure 6:** Multivariate logistic analysis results and risk factor scores.

**Figure 7:** Diagnostic efficacy of ultrasound signs of malignant thyroid nodules.

**Figure 8:** Sensitivity and specificity of different diagnostic cutoff points of CEUS.

**Table 1:** Comparison of the general data of benign and malignant thyroid nodules.

Project	Normal information	Malignant	Benign	*X* ^2^	*P* value
Gender	Female	77.5	84.3	0.422	0.526
	Male	21.6	15.8		

Age	＜42 years old	40.3	31.9	1.289	0.557
	42–70 years old	56.7	63.2		
	≥70 years old	2.8	5.8		

Background	Normal	92.4	88.76	0.884	0.36
	Abnormal	4.8	11.2		

Number of nodules	Single shot	36.8	26.3	0	1
	Multiple shots	73.2	73.4		

RETRACTED

**Table 2:** Comparison of different ultrasound signs in differentiating benign and malignant nodules.

Project	Ultrasound signs	Malignant (%)	Benign (%)	*X*^2^ value	*P* value
Ingredient	Reality	100	69.8	15.096	≤0.001
	Cysticity	0	30.2		

Echo type	Low echo	87.8	44.5	24.389	≤0.001
	Wait for echo	12.2	55.7		

Texture	Even	14.6	24.3	1.257	0.261
	Uneven	85.7	76.1		

Form	Rule	39.3	84.9	48.198	≤0.001
	Irregular	61.2	12.5		

Aspect ratio	≥1	58.3	5.9	76.277	≤0.001
	<1	41.5	94.3		

Calcification	No	25.6	72.5	43.302	≤0.001
	Microcalcification	41.3	11.2		
	Coarse calcification	33.1	16.8		

Edge	Clear	39.2	82.5	33.813	≤0.001
	Not clear	61.5	17.3		

Coating	Envelope invaded	34.2	6.8	31.514	≤0.001
	Good coating	65.9	93.2		

**Table 3:** Contrast enhancement mode of thyroid nodules.

Pathological type	Nodular goiter	Atypical follicular adenoma	Papillary carcinoma	Total
Quantity	18	2	17	37
Low enhancement	3	2	12	17
Equal enhancement	5	6	6	17
High enhancement	9	2	3	14
Uneven enhancement	5	2	5	12

**Table 4:** CEUS enhancement mode and pathological comparison results.

Grouping	Divide	Malignant	Benign	*X* ^2^	*P*
Distribution	Even	10	16	3.868	0.041
	Uneven	36	27		

Degree of enhancement	High enhancement	4	4	6.035	0.049
	Equal enhancement	3	10		
	Low enhancement	42	28		

Boundary	Clear	22	29	4.167	0.033
	Blurry	28	15		

Range	Narrow	12	5	3.051	0.071
	Constant	38	38		

Enhancement direction	Radial	18	7	4.289	0.034
	Dispersion	32	36		

Perfusion time	Fast-forward	4	2	24.235	≤0.001
	Synchronize	15	28		
	Back	27	13		

**Table 5:** Consistency results of TI-RADS descriptors for physicians of different years.

Index	Microcalcification	Aspect ratio ≥1	Internal blood flow	Low echo	Blurred borders	Irregular shape	Reality
A	39	36	25	81	28	39	85
B	0	4	10	3	9	16	4
C	10	6	3	1	11	11	1
D	42	45	54	3	44	27	1
E	36	24	28	5	9	12	3
*K* value	0.784	0.787	0.683	0.578	0.549	0.411	0.264
*P*	0.005	<0.001	<0.001	<0.001	<0.001	<0.001	<0.001

**Table 6:** Multivariate logistic analysis results and risk factor scores.

Index	Reality	Low echo	Very low echo	Aspect ratio ≥1	Unclear boundary	Irregular shape	Microcalcification
*β*-Value	0.968	1.268	1.941	1.493	1.044	2.357	2.683
Wald *x*^2^	8.627	42.504	14.325	22.952	8.459	44.106	12.640
*P* value	0.003	<0.001	<0.001	<0.001	<0.001	<0.001	<0.001
OR value	2.645	3.533	6.958	4.146	2.846	10.515	14.598
Scoring system	10.0	13.0	20.0	15.8	10.8	24.4	27.81
Lower limit	1.382	2.416	2.548	2.425	1.415	8.262	9.182
Upper limit	5.037	5.148	19.008	8.188	5.718	9.185	23.198

RETRACTED

**Table 7:** Diagnostic efficacy of ultrasound signs of malignant thyroid nodules.

Ultrasound signs	Sensitivity	Specificity	Positive predictive value	Negative predictive value	Accuracy	Positive likelihood ratio	Odds ratio
Microcalcification	51.23	88.87	45.66	88.78	83.08	4.62	10.661
Envelope invaded	34.25	95.12	56.02	88.81	85.72	6.99	10.089
Reality	100.00	30.23	20.73	62.29	40.98	1.43	18.352
Low echo	87.81	55.57	26.48	96.16	60.51	1.98	9.123
Irregular shape	60.99	84.55	47.18	92.49	83.45	4.91	10.994
Aspect ratio ≥1	58.55	94.23	64.88	92.56	88.73	10.14	23.024
Far field	48.77	90.22	47.63	90.63	83.82	4.98	13.031
Unclear edges	60.98	83.67	39.16	92.08	73.32	3.53	7.453

**Table 8:** Sensitivity and specificity of different diagnostic cutoff points of CEUS.

Diagnostic cutoff point	Sensitivity	Specificity	Youden's index	Sen	Spe	1 − Spe
14.2	0.954	0.819	0.762	0.479	0.977	0.024
19.3	0.954	0.811	0.763	0.814	0.884	0.118
24.5	0.882	0.931	0.819	0.817	0.675	0.339
16.59	0.883	0.934	0.811	0.917	0.856	0.722
28.06	0.878	0.936	0.814	0.845	0.754	0.546
29.12	0.876	0.932	0.813	0.823	0.289	0.516
22.45	0.856	0.928	0.807	0.819	0.314	0.428

## Data Availability

No data were used to support this study.
